The article "miR-214-3p Attenuates Sepsis-Induced Myocardial Dysfunction in Mice by Inhibiting Autophagy through PTEN/AKT/mTOR Pathway" was published in 2020. Journal: Biomed Res Int.

# miR-214-3p Attenuates Sepsis-Induced Myocardial Dysfunction in Mice by Inhibiting Autophagy through PTEN/AKT/mTOR Pathway

**DOI:** 10.1155/2020/1409038

**Published:** 2020-07-02

**Authors:** Zhenzhen Sang, Pu Zhang, Yunxia Wei, Shimin Dong

**Affiliations:** ^1^Emergency Department, The Third Hospital of Hebei Medical University, No. 139 Ziqiang Road, Qiaoxi Qu, Shijiazhuang City 050051, China; ^2^Emergency Department, Cangzhou Central Hospital, No. 16 Xinhua Road, Yunhe Qu, Cangzhou City 061001, China

## Abstract

*Aims*. More than half of the patients with sepsis would develop cardiac dysfunction, which is termed as sepsis-induced myocardial dysfunction (SIMD). Previous studies suggest that autophagy may play an important role in SIMD. The present study investigated whether miR-214-3p could attenuate SIMD by inhibiting autophagy. *Main Methods*. In this article, we investigated the role of autophagy in a mouse model of cecal ligation and puncture (CLP). The structure and function of hearts harvested from the mice were evaluated. Myocardial autophagy levels were detected with immunohistochemical, immunofluorescent, and Western blot. *Key Findings*. miR-214-3p can alleviate SIMD in septic mice by inhibiting the level of cardiac autophagy to attenuate myocardial dysfunction. Moreover, this study showed that miR-214-3p inhibited autophagy by silencing PTEN expression in the myocardial tissues of septic mice. *Significance*. This study showed that miR-214-3p attenuated SIMD through myocardial autophagy inhibition by silencing PTEN expression and activating the AKT/mTOR pathway. The present findings supported that miR-214-3p may be a potential therapeutic target for SIMD.

## 1. Introduction

Sepsis, which is characterised by a systemic inflammatory response syndrome, complications with multiple organ dysfunctions, and high incidence and mortality rates, is a leading cause of death in patients with severe infection worldwide [1]. Sepsis-induced myocardial dysfunction (SIMD) is an identified serious component of the sepsis-induced multiorgan failure, and it is associated with adverse outcomes and higher mortality [2]. But the mechanisms that underlie sepsis-induced cardiomyopathy are not well-known. Autophagy is a highly regulated bulk degradation pathway to remove damaged organelles including mitochondria from the cellular milieu, and thus preserve cellular homeostasis and survival [3]. However, excessive autophagy may exert adverse effects on cardiac function and cellular health [4]. Therefore, a moderate level of autophagy is the key to reduce SIMD. miR-214 has been demonstrated to be protective for H_2_O_2_-induced cardiac myocyte injury [5] and sepsis-induced apoptosis of cardiomyocytes [6]. Recently, one study has reported that miR-214-3p could play a protective role in Alzheimer's disease by inhibiting neurons autophagy [7]. However, whether miR-214 could regulate myocardial autophagy in septic mice remains unknown. In this study, we investigated the effect and mechanism of miR-214-3p in SIMD in the CLP-treated mice model.

The article "miR-214-3p Attenuates Sepsis-Induced Myocardial Dysfunction in Mice by Inhibiting Autophagy through PTEN/AKT/mTOR Pathway" was published in 2020. Journal: Biomed Res Int.

## 2. Materials and Methods

### 2.1. Sepsis Animal Model

Six- to 8-week-old male mice (Kunming mice: the Medical Laboratory Animal Centre of the Hebei Medical University, Shijiazhuang, Hebei, China) were used in the experiments. All mice were acclimated to a 12 h day-and-night cycle under specific pathogen-free conditions with food at least 1 week before the experiments. A sepsis model was established via CLP, as previously described [8]. The mice were anesthetised by isoflurane inhalation (induced at 3% and maintained at 0.5%) using a small animal ventilator. The exposed cecum was ligated with two punctures using a 18-gauge needle. Then, the cecum gently extruded a small amount of feces and was placed back in its anatomical position. The sham model mice were operated similarly, but without ligating and puncturing of the cecum. The Animal Ethics Committee of Cangzhou Central Hospital (Committee for the Update of the Guide for the Care and Use of Laboratory Animals, 2017) approved the experimental protocols.

Mice (*n* = 10 for sham operation and CLP) were randomly assigned to six groups as follows: Sham group, CLP group, mimics control+CLP group, miR-214-3p mimics+CLP group, inhibitor control+CLP group, and miR-214-3p inhibitor+CLP group. The Sham group mice were exposed to the same procedure but without ligation and puncture of the cecum. Mice in the other groups received cecal ligation and perforation. Twenty-four hours after the last treatment, all mice were quickly anesthetized with chloralic hydras to collect blood and heart samples.

### 2.2. In Vivo Transfection

The mice were transfected with miR-214-3p mimics–mimics control or miR-214-3p inhibitor–inhibitor control using adenovirus (2 × 10^11^pfu) (GenePharma, Shanghai, China) for 4 days according to the manufacturer's protocol. The mice were anesthetised, and 200*μ*l adenovirus was injected into tail veins.

### 2.3. Cardiac Injury Marker Detection

The mice in each group were killed at 6, 12, and 24 h post-CLP. Blood samples were harvested from mice heart, followed by centrifugation for collecting serum. The serum levels of creatine kinase–MB (CK–MB) and lactate dehydrogenase (LDH) were determined using an automated analyser (Abbott Architect, Abbot Park, Illinois, USA).

### 2.4. Echocardiography Measurements

Cardiac function parameters, such as left ventricular structure and function, were also assessed via echocardiography [9]. In the vivo imaging system, echocardiographic measurements were taken using a Vevo 2100 high-resolution (Visual Sonics Inc., Toronto, Canada). The left ventricle ejection fraction (LVEF, %) and fraction shortening (FS, %) were measured and assessed as indicators of cardiac function.

The article "miR-214-3p Attenuates Sepsis-Induced Myocardial Dysfunction in Mice by Inhibiting Autophagy through PTEN/AKT/mTOR Pathway" was published in 2020. Journal: Biomed Res Int.

### 2.5. Real-Time Polymerase Chain Reaction (RT-PCR)

The mice in each group were killed at 24 h post-CLP. Total RNA was extracted from cardiac tissues via the trizol method and reverse transcribed using a one-step RT-PCR kit (GeneCopoeia, USA). miRNA levels were normalized to U6 small nuclear RNA. The sequences of the primers used are presented as follows: miR-214-3p forward, 5′- GTC GTA TCC AGT GCA GGG TCC GAG GTA TTC GCA CTG GAT ACG ACA CTG CC-3′ and reverse, 5′-GCA CAG CAG GCA CAG ACA-3′; U6 (internal control) forward, 5′-CTC GCT TCG GCA GCA CA-3′ and reverse, 5′-AAC GCT TCA CGA ATT TGC GT-3′; NLRP3 forward, 5′- CCA TCG ATA TGA CGA GTG TCC GTT GC-3′ and reverse, 5′- CCG CTC GAG CTA CCA GGA AAT CTC GAA GAC-3′.

### 2.6. Cardiac Histological Analysis

Mice were killed at 24 h post-CLP. Hearts fixed in 4% paraformaldehyde were dehydrated, seeded, dipped in wax, embedded, sectioned, and stained with hematoxylin and eosin stain and then observed by light microscopy (Olympus, Japan).

### 2.7. Transmission Electron Microscopy (TEM)

Mice were killed at 24 h post-CLP. After the fresh cardiac tissues of the left ventricle were obtained, then transmission electron microscopy was performed as described previously [10]. The samples after pretreatment were cut into thin sections (60–70 nm). The observation was done on a transmission electron microscope (Tecnai, Hitachi, Tokyo, Japan) at 80 kV Electron Microscopy Film 4489 (Kodak, ESTAR thick base, San Francisco, CA).

### 2.8. Immunofluorescent and Immunohistochemical Analysis

The fresh cardiac tissues were placed in 15% sucrose in PBS at 4°C for 4 hrs. These tissues were then exchanged for 30% sucrose in PBS, and incubation continued at 4°C overnight. The cardiac tissues were frozen in optimum cutting temperature compound and sectioned serially into sections (7 *μ*m) using a cryostat. For immunofluorescence, the sections were stained using LC3 (1 : 500). All fluorescence images were digitally acquired using a fluorescence microscope (Keyence Co, Japan).

The fresh cardiac tissues were fixed in 4% paraformaldehyde and were embedded in paraffin. The paraffin-embedded myocardial tissues were sectioned and incubated with a monoclonal antibody for the p62 (1 : 400) protein. Positive staining (brown yellow) was identified under a light microscope (Olympus, Japan). The intensity of positive staining was determined using Image pro plus 6.0 image analysis software. The integral optical density (IOD) was calculated to represent the intensity. IOD values increased as protein expression increased.

The article "miR-214-3p Attenuates Sepsis-Induced Myocardial Dysfunction in Mice by Inhibiting Autophagy through PTEN/AKT/mTOR Pathway" was published in 2020. Journal: Biomed Res Int.

### 2.9. Western Blot

Western blot analysis was performed in accordance to standard protocols. Total proteins were prepared from mice hearts. Total protein extracts were isolated from mice hearts with 250 mM sucrose buffer. Primary antibodies against AKT (1 : 1000), p-AKT (Ser-473, 1 : 1000), mTOR (1 : 1000), p-mTOR (Ser2448, 1 : 1000), PTEN (1 : 1000), p62 (1 : 1000), LC3-II/I (1 : 1000), STAT3, p-STAT3 (Ser-727, 1 : 1000), and *β*-actin (1 : 2000) were purchased from Cell Signalling Technology (Beverly, MA). Band images were scanned, and densitometric analysis was performed using NIH Image software (Bethesda, MD, USA).

### 2.10. Statistical Analysis

All values are expressed as the means ± SD and were analysed using GraphPad Prism software 8.01 (GraphPad Software Inc., San Diego, CA, USA). When only two groups were compared, an unpaired *T*-test was used. Differences were evaluated by one-way analysis of variance (ANOVA; three or more groups). *P* < 0.05 was considered statistically significant.

## 3. Results

### 3.1. Overexpression of miR-214-3p Attenuates Mortality Rate

The septic mice exhibited 30% mortality at 24 h post-CLP surgery. However, mortality rates in miR-214-3p mimics group and miR-214-3p inhibitor group were 20% and 40% at 24 h post-CLP surgery, respectively. Overexpression of miR-214-3p significantly reduced the 24 h mortality in septic mice, while inhibition of miR-214-3p increased the mortality. In contrast, their respective control oligos had no effect on mortality compared with CLP mice.

### 3.2. CLP Induces Cardiac Injury and miR-214-3p Upregulation in Cardiac Tissues

Our investigation shows that CLP decreased LVEF and FS, which is considerable on SIMD in mice at 6 h post-CLP surgery. On the contrary, the septic mice showed that myocardial enzyme indicators (e.g., LDH and CK-MB) were increased at 12 h post-CLP surgery. In addition, the expression of miR-214-3p was significantly higher in septic mice than in sham mice at 24 h post-CLP surgery (1.52-fold, *P* < 0.001, Figure 1(a)). Moreover, to explore the role of miR-214-3p in SIMD, we increased miR-214-3p expression by miR-214-3p mimic–mimic control in septic mice, while we decreased miR-214-3p expression by miR-214-3p inhibitor–inhibitor control. In Figure 1(b), 4 days after the mice were transfected with miR-214-3p mimics or inhibitor, miR-214-3p mimics increased miR-214-3p expression by 3.64-fold (*P* < 0.001), and miR-214-3p inhibitor decreased by 79.8% in cardiac tissues compared with CLP mice (*P* < 0.001). In contrast, their respective control oligos had not effect on miR-214-3p expression compared with CLP mice (*P* > 0.05).

The article "miR-214-3p Attenuates Sepsis-Induced Myocardial Dysfunction in Mice by Inhibiting Autophagy through PTEN/AKT/mTOR Pathway" was published in 2020. Journal: Biomed Res Int.

### 3.3. Overexpression of miR-214-3p Attenuates Myocardial Dysfunction in Septic Mice

To verify whether the overexpression of miR-214-3p could attenuate the damage of cardiac function caused by sepsis, the septic mice underwent CLP surgery, and echocardiography measurements were further performed subsequently. At 6 h post-CLP surgery, LVEF and FS varied most notably. Thus, we observed the cardiac function of each group. As shown in Figures 2(a) and 2(b), LVEF and FS were significantly decreased in septic mice than in sham mice at 6 h post-CLP surgery (All *P* < 0.001), as measured by echocardiography. However, mice transfected with miR-214-3p mimics showed a significant increase of LVEF and FS compared to the CLP group (All *P* < 0.001), while transfected with miR-214-3p inhibitor showed significant decrease of LVEF and FS (All *P* < 0.001). In contrast, their respective control oligos had no effect on the value of LVEF and FS compared with CLP mice (*P* > 0.05). This result indicated that the overexpression of miR-214-3p could improve myocardial function, which was decreased by CLP surgery (Figures 2(a) and 2(b)).

### 3.4. Overexpression of miR-214-3p Attenuates Myocardial Injuries in Septic Mice

To detect the myocardial function of CLP-induced sepsis, serum LDH and CK-MB levels were measured at 12 h post-CLP surgery. In Figures 2(c) and 2(d), the serum LDH and CK-MB levels significantly increased after CLP surgery compared with the sham mice (*P* < 0.001). However, miR-214-3p mimics reduced the levels of LDH and CK-MB in the CLP group (All *P* < 0.001). The inhibition of miR-214-3p displayed an opposite tendency to the above indicators (All *P* < 0.001). Compared with CLP mice, their respective control oligomers had no effect on serum LDH and CK-MB levels (*P* > 0.05). The results showed that the overexpression of miR-214-3p attenuate myocardial injury in septic mice.

### 3.5. Overexpression of miR-214-3p Attenuates Myocardial Pathological Damage

The histological analysis of the heart tissues from CLP-treated mice showed myocardial necrosis and interstitial edema adjacent to localized extravasation of red blood cells compared with sham-operated mice, which were normal. These pathological changes were significantly attenuated by the overexpression of miR-214-3p, while aggravated by the inhibition of miR-214-3p (Figure 3).

Moreover, myocardial histopathological changes were observed via TEM. As shown in Figure 4, myocardial tissues from the sham-operated mice showed normal structure with proper mitochondria distribution, while CLP mice revealed cellular disorganisation, myofibrillar disarray larger autophagosomes and more autolysosomes. The overexpression of miR-214-3p attenuates myocardial histopathological changes in septic mice whilst aggravating the inhibition of miR-214-3p mice. In contrast, their respective control oligos had no effect on the myocardial histopathological changes (Figure 4).

The article "miR-214-3p Attenuates Sepsis-Induced Myocardial Dysfunction in Mice by Inhibiting Autophagy through PTEN/AKT/mTOR Pathway" was published in 2020. Journal: Biomed Res Int.

### 3.6. Overexpression of miR-214-3p Inhibits Myocardial Autophagy in Septic Mice

LC3 is a maker of autophagy, and LC3-II/I ratio could be viewed as a ruler to estimate autophagy. In addition, p62 is often used as an index of autophagic flux. The hearts were sliced for myocardial tissue biopsy, then several autophagic assay methods were performed.

Firstly, we examined the changes in the LC3 in cardiac tissues using immunofluorescence staining. In Figure 5, in the sham group, LC3 red fluorescence showed diffuse distribution and did not form bright fluorescent dots, whereas in the CLP group, the bright red dots were evidently aggravating around in the cytoplasm (*P* < 0.001), which was a sign of autophagy. Immunofluorescence staining results showed that the overexpression of miR-214-3p reduced the fluorescence intensity of LC3 in cardiac tissues (*P* < 0.001), suggesting that the overexpression of miR-214-3p inhibited autophagy. However, the inhibition of miR-214-3p displayed an opposite result (*P* < 0.001). In contrast, their respective control oligos had no effect on the changes in the LC3 in cardiac tissues (*P* > 0.05, Figure 5).

Secondly, we examined the changes in p62 in cardiac tissues using immunohistochemistry staining. In Figure 6, the p62 in the sham group was strongly positive because it was normally accumulated without autophagy. As expected, the number of p62 decreased significantly in the CLP group because of the activated autophagy compared with the sham group (*P* < 0.001). The expression level of p62 was lower in the miR-214-3p mimic group and higher in the miR-214-3p inhibitor group compared with the CLP group (All *P* < 0.001). In contrast, their respective control oligos had no effect on the changes in p62 in cardiac tissues (*P* > 0.05, Figure 6).

Thirdly, we examined the changes in LC3 and p62 in cardiac tissues using Western blot analysis. In Figure 7(a), CLP significantly increased the rate of LC3-II/LC3-I but significantly decreased the levels of p62 (All *P* < 0.001), indicating that sepsis induced myocardial autophagy. Overexpression of miR-214-3p decreased LC3-II/LC3-I ratio whilst increasing p62 levels (All *P* < 0.001). However, the inhibition of miR-214-3p displayed an opposite tendency to the above indicators (All *P* < 0.001), further confirming the suppressive effect of miR-214-3p on mice myocardial autophagy. In contrast, their respective control oligos had no effect on the changes in the rate of LC3-II/LC3-I and the levels of p62 in cardiac tissues (*P* > 0.05, Figure 7(a)). Results showed that autophagy was induced by CLP, and the overexpression of miR-214-3p could partially inhibit it.

The article "miR-214-3p Attenuates Sepsis-Induced Myocardial Dysfunction in Mice by Inhibiting Autophagy through PTEN/AKT/mTOR Pathway" was published in 2020. Journal: Biomed Res Int.

### 3.7. Overexpression of miR-214-3p Inhibits Myocardial Inflammation in Septic Mice

As shown in Figure 8, the expression of NLRP3 was significantly higher in septic mice than in sham mice at 24 h post-CLP surgery. However, miR-214-3p mimics reduced the expression level of NLRP3 in septic mice (All *P* < 0.001). The inhibition of miR-214-3p displayed an opposite tendency to the expression of NLRP3 (All *P* < 0.001). Compared with CLP mice, their respective control oligomers had no effect on the level expression of NLRP3 (*P* > 0.05). The results showed that the overexpression of miR-214-3p attenuate myocardial inflammation in septic mice.

### 3.8. Overexpression of miR-214-3p Activates the AKT/mTOR Signalling Pathway to Inhibit Autophagy via Silencing of PTEN in Cardiac Tissues

It is well-acknowledged that PTEN/AKT/mTOR is an important signaling pathway regulating autophagy, and PTEN is a negative inhibitor of the AKT/mTOR signalling pathway. To investigate the effect of miR-214-3p on the PTEN-AKT/mTOR pathway, the protein levels of AKT, mTOR, and PTEN were analysed through Western blot analysis. In Figure 7(b), CLP significantly decreased the expression of p-AKT and p-mTOR (All *P* < 0.001), but significantly increased the PTEN levels (*P* < 0.001). The overexpression of miR-214-3p decreased the PTEN levels whilst increasing p-AKT and p-mTOR levels (All *P* < 0.001). However, the inhibition of miR-214-3p displayed an opposite tendency to the above indicators (All *P* < 0.001). In contrast, their respective control oligos had no effect on the PTEN-AKT/mTOR pathway in cardiac tissues (*P* > 0.05, Figure 7(b)). Our results suggested that sepsis inhibits the PTEN-AKT/mTOR pathway. The overexpression of miR-214-3p activated AKT/mTOR pathway via the silencing of PTEN in cardiac tissues.

### 3.9. Overexpression of miR-214-3p Suppressed the Expression of STAT3 in Cardiac Tissues

The signal transduction and activator of transcription 3 (STAT3), one of the seven STAT family members, is a bifunctional protein which involved in signal transduction via tyrosine phosphorylation in the cytoplasm. In Figure 9, CLP significantly decreased the expression of p-STAT3 (*P* < 0.001). The overexpression of miR-214-3p induced a significant increase of p-STAT3 (*P* < 0.001). However, the inhibition of miR-214-3p significantly decreased the expression of p-STAT3 (*P* < 0.001). In contrast, their respective control oligos had no effect on the expression of p-STAT3 in cardiac tissues (*P* > 0.05, Figure 9).

The article "miR-214-3p Attenuates Sepsis-Induced Myocardial Dysfunction in Mice by Inhibiting Autophagy through PTEN/AKT/mTOR Pathway" was published in 2020. Journal: Biomed Res Int.

## 4. Discussion

Autophagy is a highly regulated bulk degradation mechanism for the intracellular clearance of long-lived proteins and the recycling of cytoplasmic contents [11]. However, autophagy is believed to play a “double-edged sword” role in the maintenance of cardiovascular homeostasis. In this report, a SIMD model was established by CLP surgery to investigate the function of miR-214-3p. Firstly, the overexpression of miR-214-3p significantly alleviated myocardial dysfunction and myocardial injuries in septic mice. Secondly, miR-214-3p protects cardiomyocytes from sepsis-induced injuries via the inhibition of myocardial autophagy. Thirdly, the protective effect of miR-214-3p may be related to the activation of the AKT/mTOR signalling pathway to inhibit autophagy in cardiomyocytes via silencing PTEN.

In our study, we prepared a sepsis model using CLP surgery to investigate the pathogenesis of SIMD, which is a classic animal model of sepsis [8]. In CLP mice, the cardiac injury markers of serum LDH and CK-MB levels and the echocardiography of LVEF and FS showed that CLP leads to SIMD. Also, the CLP mice presented myocardial histopathological changes. As expected, the overexpression of miR-214-3p significantly attenuated myocardial injuries and myocardial dysfunction of SIMD. However, the inhibition of miR-214-3p displayed an opposite tendency to the above indicators.

NLRP3 represents one of the most comprehensively characterized inflammasomes that was shown to be involved in diverse conditions such as sepsis, infectious diseases, and auto-inflammatory diseases. Excessive activation of the NLRP3 inflammasome is believed to be an important factor in the pathological development of septic injury [12]. In our study, the expression of NLRP3 was significantly higher in septic mice than in sham mice at 24 h post-CLP surgery. However, miR-214-3p mimics reduced the expression level of NLRP3 in septic mice (*P* < 0.001). The result showed that the overexpression of miR-214-3p attenuates myocardial inflammation in septic mice.

Accumulated evidence revealed the regulatory effect of autophagy on sepsis-induced cardiac dysfunction [13, 14]. Previous studies have shown that a complete autophagy is a highly dynamic process, which is represented as autophagic flux characterized by the autophagosomal formation and maturation via fusion with lysosomes [15]. However, the role of autophagy in the heart has been controversial, low levels of autophagy are beneficial to cardiomyocytes, and excessive autophagy can cause unwanted cardiomyocyte damage [19, 20]. Hence, keeping moderate levels of autophagy is the key to attenuate myocardial injury in septic condition. It was shown that autophagy was activated initially in sepsis, followed by a subsequent phase of dysfunction due to autophagic cell death [16]. Furthermore, it has been identified that the inhibition of autophagy is cardioprotective against sepsis-induced myocardial injury [17–19]. It has been reported that autophagy can be both a protective process and a precursor to cell death depending on the intensity and duration of the insult [20]. The autophagic process requires completion of all steps of the process, to result in digestion of dysfunctional proteins or organelles. And impairment of the autophagic process contributes to cardiac dysfunction during sepsis [20]. Hence, keeping moderate levels of autophagy is the key to attenuate myocardial injury in septic condition. In this study, our results indicate that the autophagy process was completed and accelerated in CLP mice. The overexpression of miR-214-3p could significantly inhibit CLP-induced autophagy in myocardial tissues, which was proven by the change in protein markers, such as LC3-II/I and p62, as well as a significant increase in autophagosomes. However, the inhibition of miR-214-3p displayed an opposite tendency to the aforementioned indicators. The results of immunofluorescence and immunohistochemistry after CLP surgery also provided further evidence that the overexpression of miR-214-3p inhibited autophagy in myocardial tissues. Moreover, accumulating evidences have indicated that the overexpression of miR-214 could inhibit autophagy in various cells and tissues [7, 21, 22]. Our results demonstrated that the overexpression of miR-214-3p attenuates CLP-induced myocardial injury by inhibiting excessive autophagy.

The article "miR-214-3p Attenuates Sepsis-Induced Myocardial Dysfunction in Mice by Inhibiting Autophagy through PTEN/AKT/mTOR Pathway" was published in 2020. Journal: Biomed Res Int.

Notably, PTEN/AKT/mTOR is an important signalling pathway that regulates myocardial autophagy, which plays a key role in heart diseases [14, 23]. PTEN is a negative inhibitor of the AKT/mTOR signalling pathway [24]. Yang et al. [25] reported that miRNA-214 suppresses oxidative stress in diabetic nephropathy via the ROS/Akt/mTOR signaling pathway and uncoupling protein2. Liu et al. reported that miR-214 could regulate autophagy through the PI3K/AKT signalling pathway in the rat model of myocardial fibrosis [26]. Gong et al. reported that Oridonin relieved hypoxia-caused apoptosis and autophagy via adjusting the PI3K/AKT/mTOR pathway through the enhancement of miR-214 in H9C2 cells. Additionally, PTEN was forecasted to be a first-hand target of miR-214 [27]. Hu et al. reported that miR-214 promotes radio sensitivity by the inhibition of ATG12-mediated autophagy in colorectal cancer (CRC). Importantly, miR-214 is a determinant of CRC irradiation response and may serve as a potential therapeutic target in CRC treatment [28]. Therefore, we hypothesised that the effects of miR-214-3p in CLP-treated mice might be involved in the regulation of the PTEN/AKT/mTOR pathway. Interestingly, our results showed that CLP significantly elevated the levels of PTEN but decreased the levels of p-AKT and p-mTOR, indicating that CLP inactivated the AKT/mTOR pathway. Furthermore, the overexpression of miR-214-3p decreased the PTEN levels whilst increasing p-AKT and p-mTOR levels (*P* < 0.001). However, the inhibition of miR-214-3p displayed an opposite tendency to the above indicators (*P* < 0.001). These data support miR-214-3p as an activator of the AKT/mTOR pathway by the silencing of PTEN, which emphasised and confirmed the similar myocardial protective effect of miR-214-3p in SIMD.

It has been reported that the inhibition of autophagy contributes to the accumulation and immunosuppressive function of myeloid-derived suppressor cells (MDSCs) by promoting the activation of STAT3 signaling in endotoxin shock [29]. STAT3 has been reported that in protected hearts, its phosphorylation is necessary for mitochondrial localization. STAT3 activation as a central point [30], the activation/phosphorylation of several kinases (e.g., AKT, ERK1/2, GSK3b) was promoted. Previous research reported that STAT3 is able to bind to the promoter region of miR-214 [31]. miR-214 can modulate the downstream PTEN/(PI3K)/AKT/mTOR signalling pathways. Interestingly, our results showed that the overexpression of miR-214-3p induced a significant increase of p-STAT3. Therefore, combined with the experimental results, we speculated that STAT3 may be an upstream target of miR-214, whose activation can inhibit autophagy together with miR-214 through the AKT/mTOR signaling pathway. Further studies are needed to accurately determine the effects of autophagy on the accumulation and functional activity of STAT3 by using shRNA, which are very important for autophagy in vitro and miR-214 knockout mice in vivo.

## 5. Conclusions

In conclusion, this study uncovered a potential mechanism underlying the protective role of miR-214-3p against SIMD involving the inhibition of autophagy through the PTEN/AKT/mTOR pathway. The present findings support that miR-214 may be a potential therapeutic target for SIMD. Although we used autophagy mechanisms to establish the influence of miR-214-3p in SIMD, clinical evidence is necessary to support our findings further.

The article "miR-214-3p Attenuates Sepsis-Induced Myocardial Dysfunction in Mice by Inhibiting Autophagy through PTEN/AKT/mTOR Pathway" was published in 2020. Journal: Biomed Res Int.

## Figures and Tables

**Figure 1:** Relative miR-214-3p expression (a) CLP increased miR-214-3p expression in myocardial tissue detected by qRT-PCR. (b) miR-214 expression through the injection of miR-214-3p mimics increased by 3.64-fold and with miR-214-3p inhibitor decreased by 79.8% in mice hearts compared with CLP-treated mice at 24 h. ^$^*P* < 0.01, significantly different from Sham, ^#^*P* < 0.01, significantly different from CLP (*n* = 3 per group).

**Figure 2:** Overexpression of miR-214-3p attenuates myocardial injuries in septic mice. (a) Effect of miR-214-3p mimics on cardiac function parameter LVEF. (b) Effect of miR-214-3p mimics on cardiac function parameter FS. (c) Effect of miR-214-3p mimics on serum LDH in mice. (d) Effect of miR-214-3p mimics on serum CK-MB in mice. ^$^*P* < 0.01 compared with sham, ^#^*P* < 0.01 compared with CLP (*n* = 6 per group).

**Figure 3:** Overexpression of miR-214-3p attenuates histological changes in the myocardial tissues at 24 h post-CLP (haematoxylin-eosin, ×400). Scale bar, 50 *μ*m.

**Figure 4:** Overexpression of miR-214-3p attenuates myocardial autophagy caused by CLP. Transmission electron microscopy (TEM) images of myocardial tissues at 24 h post-CLP (×15000).

**Figure 5:** Immunofluorescence expression of LC3 was quantified by fluorescence intensity (×200). Scale bar, 50 *μ*m, ^$^*P* < 0.01 compared with sham, ^#^*P* < 0.01 compared with CLP (*n* = 6 per group).

**Figure 6:** Immunohistochemistry expression of p62 was quantified by IOD (×400). Scale bar, 20 *μ*m, ^$^*P* < 0.01 compared with sham, ^#^*P* < 0.01 compared with CLP (*n* = 6 per group).

**Figure 7:** Overexpression of miR-214-3p inhibits myocardial autophagy and autophagy-related signal pathways. (a) Effect of miR-214-3p on autophagy markers LC3 and p62 along with control protein *β*-actin. (b) Effect of miR-214-3p on the autophagy-related signal pathway. ^$^*P* < 0.01 compared with sham, ^#^*P* < 0.01 compared with CLP (*n* = 3 per group).

**Figure 8:** Relative NLRP3 expression. CLP increased the expression level of NLRP3 in myocardial tissue detected by qRT-PCR. miR-214-3p mimics reduced the expression level of NLRP3, while miR-214-3p inhibitor increased the expression level of NLRP3 compared with CLP-treated mice at 24 h. ^$^*P* < 0.01, significantly different from Sham, ^#^*P* < 0.01, significantly different from CLP (*n* = 6 per group).

**Figure 9:** Overexpression of miR-214-3p suppressed the expression of STAT3 in cardiac tissues. ^$^*P* < 0.01 compared with sham, ^#^*P* < 0.01 compared with CLP (*n* = 3 per group).

## Data Availability

The data used to support the findings of this study are included within the article.

The article "miR-214-3p Attenuates Sepsis-Induced Myocardial Dysfunction in Mice by Inhibiting Autophagy through PTEN/AKT/mTOR Pathway" was published in 2020. Journal: Biomed Res Int.

## Abbreviations

CLP: Cecal ligation and puncture
SIMD: Sepsis-induced myocardial dysfunction.
